# Computer Added Simulation of the Spread of Multidrug-Resistant Bacteria in an Radiation Therapy Shelter Based on Computational Fluid Dynamics

**DOI:** 10.1155/2022/4760823

**Published:** 2022-07-06

**Authors:** Kuan Wu, Xiadong Li, Xiaoyan Miu, Huichun Feng

**Affiliations:** ^1^Department of Tumor Radiotherapy, First People's Hospital of Fuyang, 311400 Hangzhou, China; ^2^Department of Tumor Radiotherapy, Hangzhou First People's Hospital, Wushan District, 310000 Hangzhou, China

## Abstract

**Purpose:**

Due to the poor ventilation and air stagnation in the radiation therapy ward, it is easy to cause respiratory disease transmission, which brings about the public health safety problem of infection. In order to alleviate this problem, we propose a research method based on computational fluid dynamics (CFD).

**Method:**

A three-dimensional model of a radiation therapy ward is established, and the CFD software framework is used to numerically simulate the air flow field in the constrained radiation therapy ward environment. We computed the influence of the spray speed, particle size, and inlet content of respiratory droplets on the flow and spread of multidrug-resistant bacteria.

**Results:**

In the range of the horizontal transmission line *X* from 0 to 3 meters, when the transmission speed (*V*) is 35 m/s, the multidrug-resistant bacteria concentration reaches the highest value. In the range of the vertical transmission line *Y* from 0 to 3 meters, when *V* is 35 m/s, the multidrug-resistant bacteria concentration reaches the highest value.

**Conclusion:**

A large amount of data shows that there is a positive correlation between the respiratory droplet spray velocity, inlet content, and the multidrug-resistant bacteria flow propagation speed and concentration distribution. The respiratory droplet size mainly affects the peak concentration of the multidrug-resistant bacteria flow propagation.

## 1. Introduction

Due to the impact of other airborne bacteria, organized and controlled natural ventilation should be considered in the design and planning of modern radiation therapy wards. First of all, computational fluid dynamic (CFD) technology must be applied to the wind environment around the radiation therapy ward and the radiation therapy ward interior during the design phase [1–4]. Detailed analysis is as follows: secondly, a controlled natural ventilation structure can be used in the radiation therapy ward. For example, the breathing wall technology frequently used in foreign countries in recent years combines the visual effect of the glass curtain wall with the environmental function of natural ventilation [5–7]. Opening windows for ventilation in the room avoids the disadvantages of opening windows in high-rise radiation therapy wards. At the same time, it is also a very effective energy-saving measure.

The population is generally susceptible to the multidrug-resistant bacteria [8–13]. Pneumonia caused by the new multidrug-resistant bacteria infection can occur in people with low immune function and normal immune function, and it has a certain relationship with the amount of exposure to the virus. For people with poor immune function, such as the elderly, pregnant women, people with abnormal liver and kidney function, and people with chronic diseases, the condition will be more severe after infection.

The main mode of transmission of the multidrug-resistant bacteria is through respiratory droplets, and it can also be spread through contact. The transmission process is specifically that droplets or other virus-rying body fluids are deposited on the surface of the paper. After the hand touches the pollution, it then touches the mucous membranes of the mouth, nasal cavity, and eyes, resulting in infection. Judging from the order of incidence of some clusters of cases, the characteristics of human-to-human transmission are very obvious, and there is a certain range of community transmission.

With the outbreak of the new bacteria epidemic in 2020, a large number of papers about the spread of respiratory droplets in the air appeared, which provided good guidance for our research. Bhagat et al. [14] studied the influence of radiation therapy ward ventilation on the transmission path of respiratory droplets and further proved the risk of virus transmission in the air. Mittal et al. [15] warned that the diffusion and deposition of droplets in the air are the key factors of transmission. At the same time, they also summarized the scientific significance and mechanism behind face masks, hand washing, and indoor ventilation.

Agrawal and Bhardwaj [16] have shown through research that the droplet cloud produced by coughing pollutes the air a lot, and the droplet cloud has self-similar properties, which can help people design better closed space ventilation systems. Verma et al. [17] used mobile display technology to study the effect of medical masks in reducing the speed and propagation distance of respiratory droplets and also found that there would be some small leaks at the edges of the masks, which provided an effective assessment for medical staff and mask manufacturers.

In recent years, CFD has been increasingly used to study the spread of bacteria in radiation therapy wards [18–20], which is of great significance for preventing the multidrug-resistant bacteria and improving public health safety. Taking a radiation therapy ward as the research object, we used a CFD framework to simulate the air flow field of the ward under different air supply conditions in summer and calculated according to the simulation results to obtain the respiratory droplet injection velocity, particle size, and inlet content to the droplet flow. The law of influence of transmission is analyzed, and the concentration distribution of multidrug-resistant bacteria on the horizontal transmission line and the vertical transmission line is analyzed.

## 2. Methods

### 2.1. Airflow Research Method

The current mainstream airflow research methods include multizone simulation method, experimental research method, and CFD simulation method.

Because the multizone simulation method oversimplifies the system, it will produce large errors; so, it is only suitable for predicting the ventilation of multizone radiation therapy wards with more uniform room distribution and not suitable for predicting the airflow distribution in the radiation therapy ward. The experimental research method is difficult to implement because it is often affected by the site and weather.

The CFD method relies on its powerful ability to capture microscopic flow phenomena to make up for the above research deficiencies and can predict the airflow organization (referring to the organization of airflow direction and uniformity according to certain requirements) and pollutant diffusion in confined spaces. Nielsen [21] first applied CFD to the prediction of indoor air distribution. Topp et al. [22] found that the influence of complex geometric shapes on the local calculation results is obvious. Murakami and Kato [23] used CFD to analyze the microclimate around the human body and compared the effects of different boundary conditions. Zhang and Chen [24] simulated diffusion at different ventilation rates and evaluated Euler and Lagrangian models.

### 2.2. Governing Equations and Numerical Methods

For the spread of bacteria in the air, from the perspective of fluid mechanics, it is actually a flow of very small particles in the air. The general fluid flow can be described by the vortex function analysis method; in order to use the streamline tracing technology and to simplify the complexity of the problem, the Navier-Stokes equation [25–27] of the two-dimensional viscous incompressible fluid flow is used to describe the air flow, which can be expressed in the form of infinite rigid flow function vorticity in rectangular coordinates. The Navier-Stokes equation is shown in Equations (1) and (2).

(1) ∂U∂t+∂F∂x+∂G∂y+∂H∂z=1ReL∂Fv∂x+∂Gv∂y+∂Hv∂z,

(2) $$\begin{array}{c} \rho \frac{\partial \text{y}}{\partial \text{x}}+\rho \left(v\times \nabla \right)v=-\nabla P+\rho g+\mu \nabla^{2}v, \end{array}$$

(3) $$\begin{array}{c} \nabla \times v=0. \end{array}$$

The flow was governed by the Navier-Stokes equation and continuity equation as follows:

(4) $$\begin{array}{c} \frac{\partial o}{\partial t}+w\frac{\partial o}{\partial x}+s\frac{\partial o}{\partial y}=\frac{1}{Re^{2}}o, \end{array}$$

(5) $$\begin{array}{c} \frac{\partial^{2}d}{\partial x^{2}}+\frac{\partial^{2}d}{\partial y^{2}}=-o. \end{array}$$

In Equations (4) and (5), *x* is the abscissa, *y* is the ordinate, *o* is the vortex, *d* is the flow function, and *w* and *s* are the velocity components. Equations (6) and (7) explain how the velocity component is calculated.

(6) $$\begin{array}{c} w=\frac{\partial d}{\partial y}, \end{array}$$

(7) $$\begin{array}{c} s=-\frac{\partial d}{\partial x}. \end{array}$$

### 2.3. Simulation of Flow Field in Radiation Therapy Ward

#### 2.3.1. Physical Model

We build a physical model of the station and measure the distance from the entrance to the opposite platform as the length of the station and the distance of the ward at the radiation therapy ward as the width, the *X* direction is the length of the station, the *Y* direction is the width of the station, and the *Z* direction is the height of the station. The length of the radiation therapy ward is 58.7 m, the width is 24.8 m, and the height of the roof based on the floor is 2.12 m. The physical model is shown in Figure 1. We first ignore the entire process of occupants entering the radiation therapy ward compartment. Later on, we can include human occupants as our examined model.

#### 2.3.2. Evaluation Method of Airflow Performance in Radiation Therapy Ward

When evaluating airflow performance, we need to consider the degree of uniformity of temperature and speed distribution in the station, the degree of human thermal comfort under the combined effect of airflow temperature and speed, and the energy utilization efficiency of airflow organization. We use the airflow performance evaluation index to judge the quality of the airflow organization [28, 29].

The inhomogeneity coefficient [30, 31] is a uniformity index, reflecting the performance of airflow organization and the uniformity of temperature field and velocity field distribution. The uneven coefficient can be divided into the temperature uneven coefficient *K*_*t*_ and the air velocity (wind speed) uneven coefficient *K*_*u*_.

Take *n* measuring points in the work area, measure the temperature *t*_*i*_ and the air velocity *u*_*i*_ of the measuring point *i*, and calculate the arithmetic mean *t* of temperature and the arithmetic mean *u* of air velocity at each measuring point, respectively; then, Equations (8) and (9) were as follows:

(8) $$\begin{array}{c} t=\frac{\sum t_{i}}{n}, \end{array}$$

(9) $$\begin{array}{c} u=\frac{\sum u_{i}}{n}. \end{array}$$

It can be obtained from Equations (8) and (9) that the root mean square deviation *σ_t_* of the air temperature in the radiation therapy ward and the root mean square deviation *σ_u_* of the airflow velocity are Equations (10) and (11).

(10) $$\begin{array}{c} \sigma_{t}=\sqrt{\frac{{\sum \left(t-t_{i}\right)}^{2}}{n-1}}, \end{array}$$

(11) $$\begin{array}{c} \sigma_{u}=\sqrt{\frac{{\sum \left(u-u_{i}\right)}^{2}}{n-1}}. \end{array}$$

The calculation method of the temperature unevenness coefficient *K*_*t*_ and the air velocity unevenness coefficient *K*_*u*_ are as shown in Equations (12) and (13).

(12) $$\begin{array}{c} K_{t}=\frac{\sigma_{t}}{t}, \end{array}$$

(13) $$\begin{array}{c} K_{u}=\frac{\sigma_{u}}{u}. \end{array}$$

The air distribution characteristic index (*I*_ADP_) is the percentage of the number of measuring points with the effective temperature difference within the range of -1.7 ~ 1.1°C in the working area to the total number of measuring points [32, 33]. *I*_ADP_ connects air temperature, airflow velocity, and human comfort. If *I*_ADP_ = 1, all people in the room feel comfortable; when *I*_ADP_ > 0.8, the airflow organization effect is considered satisfactory; when *I*_ADP_ ≤ 0.8, it is considered that some people feel uncomfortable, and there may be a feeling of blowing. The calculation is based on Equations (14) and (15).

(14) $$\begin{array}{c} I_{\text{ADP}}=\frac{\theta }{N}, \end{array}$$

(15) $$\begin{array}{c} \theta =\left(t_{x}-t_{r}\right)-M\left(u_{x}-u_{r}\right). \end{array}$$

In Equations (11) and (12), *θ* is the effective temperature difference, which reflects the comprehensive effect of temperature and speed. *N* is the total number of measuring points, and *t*_*x*_ is the air temperature at measuring point *x*; *t*_*r*_ is the given indoor temperature, taken as 26°C; *u_x_* is the air velocity at measuring point *x*; and *u_r_* is the air velocity in stagnation zone, taken as 0.18 m/s. It is a temperature value equivalent to the effect of unit air velocity, generally 8.56°C/(m/s).

The energy utilization coefficient *φ* can be used to evaluate the effectiveness of the energy utilization of airflow. The higher *φ* indicates the more sufficient energy utilization. The calculation method is Equation (16).

(16) $$\begin{array}{c} \varphi =\frac{t_{p}-t_{o}}{t_{n}-t_{o}}. \end{array}$$

In Equation (16), *t*_*p*_ is the exhaust air temperature, *t*_*n*_ is the average temperature of the working area, and *t*_*o*_ is the supply air temperature.

We set eight situations, and the specific characteristics of each situation are shown in Table 1.

### 2.4. The Influence of Jet Velocity

The relationship between the peak spray concentration of the inlet droplets and the number of droplets is expressed by the following Equation (14).

(17) $$\begin{array}{c} M=\frac{C}{\rho \times 1/6\times \pi \times d^{3}}. \end{array}$$

In Equation (14), *C* is the peak droplet concentration at the inlet, mg/m^3^, *M* is the number of droplets per unit volume of the inlet, 1/m^3^, *ρ* is the droplet density, kg/m^3^, and *d* is the droplet the diameter of the foam, m.

### 2.5. Measurement Configuration

A total of 70 measurement points are inserted into the radiation therapy ward configuration to measure the temperature and air speed parameters as shown in Figure 2.

## 3. Results

### 3.1. Airflow Performance Evaluation

We use numerical simulation [34–36] to perform numerical calculations on the air flow field of 8 air supply conditions. After the calculation is completed, the temperature and air velocity values of 70 measuring points are read and counted.

The suitable temperature range of the air in the radiation therapy ward in summer is 24~28°C, and the suitable air flow speed range is 0.07~0.35 m/s. Within the above range, the lower the temperature and the greater the wind speed, the better the thermal comfort of occupants. However, if the wind speed at the head position of a standing occupant exceeds 0.8 m/s, the occupant will have a strong sense of blowing.  Figure 3 shows the number of 70 measuring points satisfying suitable temperature and suitable air flow speed in 8 cases.

It can be seen from Figure 3 that the suitable temperature and air flow speed measuring points are the most in working condition (6), and the suitable air flow speed measuring points are the least in working condition (8).

From Figures 4 and 5, it can be found that in various situations, as the height of the measuring point changes from high to low, the corresponding average temperature increases, and the average wind speed decreases.

In case two, the temperature at two altitudes is the best, the wind speed at one altitude is the best, and it performs best in all working conditions. It should be pointed out that although the average temperature of the air at the height of the head of the standing occupants is lower than the minimum value of 25°C, which is suitable for all working conditions, the average wind speed at the height of occupants' feet in all working conditions is lower than the minimum value of 0.07 m/s, which is the minimum suitable air flow speed, indicating that the air circulation at this height is relatively poor. Figures 4 and 5 show that the temperature and wind speed fluctuate from high to low in the radiation therapy ward. Among them, the temperature at the height of the head of the standing occupant is lower, the wind speed is higher, and the wind speed at the height of the occupant's feet is extremely small.

It can be seen from Figure 6 that from the *I*_ADP_ data, it can be seen that the air distribution characteristics of all working conditions are relatively low, lying in the range of 30% to 50%, which is significantly lower than 80%. The fundamental reason for the low *I*_ADP_ value is the structural limitations of the train station itself and the high density of people in the radiation therapy ward.

It can be seen from the above data that only the energy utilization coefficient of case 2 is greater than 1. This shows that the system economy of the second case is the best, and its energy is fully utilized.

It can be seen from *K*_*t*_ that the *K*_*t*_ value of case 2 is the smallest and the temperature distribution is the most uniform. Through comparison, it can be found that increasing the air supply volume can significantly reduce the *K*_*t*_ value, while increasing the air supply angle can also significantly reduce the *K*_*t*_ value, and the *K*_*t*_ value decreases ratio when the air supply angle is increased from 45° to 60°. When increasing from 30° to 45°, the *K*_*t*_ value decreases greatly.

It can be seen from *K*_*u*_ that the *K*_*u*_ value of case 3 is the smallest, and the wind speed distribution is the most uniform. Through comparison, it can be found that increasing the air supply volume makes the *K*_*u*_ value significantly higher, while changing the air supply angle has little effect on the *K*_*u*_ value.

Through the above comparison and analysis of the radiation therapy ward temperature, wind speed, and airflow performance indicators under eight different air supply conditions, it can be seen that different operating conditions have their own advantages, and the indicators of the optimal operating conditions are not all the best. From the comprehensive comparison, it can be seen that the second working condition is the most ideal.

### 3.2. The Effect of Injection Speed

Figure 7 shows the multidrug-resistant bacteria concentration distribution of the horizontal transmission line and the vertical transmission line under different jet speeds. In Figure 7(a), we control *d* to 20 *μ*m, *C* to 150 mg/m^3^, *t* to 2 s, and *Y*. It is 1.6 m. When the jet velocity is 5 m/s and 15 m/s, multidrug-resistant bacteria spreads very slowly following the air flow. As the distance of *X* increases, the concentration of multidrug-resistant bacteria also decreases. When the jet velocity is 25 and 35 m/s, the distance of *X* has little effect on the concentration of multidrug-resistant bacteria.

The horizontal propagation line corresponding to each state will have a maximum concentration value, and some even have multiple maximum values. The greater the injection speed, the more concentration maximum values appear. This is a phenomenon caused by the periodic exhalation of droplets.

In Figure 7(b), we control *d* to 20 *μ*m, *C* to 150 mg/m^3^, *t* to 2 s, and *X* to 2 m. In the vertical distance, the spray speed and the multidrug-resistant bacteria concentration change pattern are consistent with the horizontal distance. When *V* reaches 35 m/s, the multidrug-resistant bacteria concentration reaches the highest value.

The spread of the virus depends very much on the ventilation air speed as it is commonly accepted that the airborne virus can be transported further in the air due to faster air flow, which can be in a multiple directions as shown in Figure 8.

In Figure 9, the simulation of the multidrug-resistant bacteria spreading from an infected occupant near the ventilation entrance is performed, and the number of healthy humans being affected is stimulated. The spread of this virus is rapid starting from the infection at the first two areas near the entrances and quickly spreading to their two neighboring areas.

## 4. Discussion

The issue of suppressing respiratory-borne diseases involves human-machine environmental engineering, public health, medicine, and other disciplines. From SARS in 2003 to multidrug-resistant bacteria in 2020, each discipline has made considerable progress in their respective fields. However, due to the latent and rapid spread of respiratory diseases, interdisciplinary exchanges and cooperation are more necessary. Many scientific issues centered on infection mechanism, prediction methods, and indoor environment design urgently need to be further studied by multidisciplinary cooperation, so as to lay a theoretical foundation for scientific infection control of respiratory tract diseases.

Although many regulations and standards propose that indoor air quality can be improved by increasing the amount of fresh air and reducing the amount of return air and thus reduce crossinfection, the above discussion is based on experience and lacks precise quantitative research.

In terms of radiation therapy ward indoor environmental engineering design, there is currently a lack of systematic research that combines indoor airflow parameters, human metabolism models, and virus diffusion laws. Research on the optimization design of air delivery and return is even rarer. How to introduce the form and parameters of ventilation into the prediction of virus spread, explain its suppression mechanism, and achieve multiobjective optimization of economy, safety, and comfort through certain algorithms are problems to be solved urgently.

Based on the concentration distribution of droplet pollutants, this paper proposes quantitative indexes when evaluating the risk of crossinfection among indoor personnel. This indicator is helpful to study the pathogenicity of droplet pollutants. On the basis of virus transmission simulation analysis, it has very important practical significance for its deepening research.

Scholars at home and abroad have laid a good foundation for the study of indoor virus aerosol droplet transmission, but they rely too much on the use of CFD simulation methods, and seldom use experimental verification, especially the use of biological for verification. Therefore, the validity of the experiment remains to be resolved.

## 5. Conclusion

This paper uses CFD to simulate and analyze the influence of different air supply conditions on the temperature, speed, and airflow performance in the radiation therapy ward. The simulation results show that, among the 8 working conditions, the air supply condition with a supply air volume of 12000 m^3^/h and an air supply angle of 60° is the optimal operating condition, and its airflow performance is better than other operating conditions. CFD-based flow field simulation can be used as an effective means to be applied to the design and optimization of radiation therapy ward ventilation systems, thereby effectively improving the thermal comfort and energy saving of wards and further affecting the spread of multidrug-resistant bacteria.

We verify the relationship between the air injection speed and the concentration of multidrug-resistant bacteria by controlling the variables, and the speed is proportional to the concentration. We must pay attention to the air supply in the radiation therapy ward, give people a better experience, reduce the probability of people catching a cold, and reduce the possibility of contracting multidrug-resistant bacteria.

## Figures and Tables

**Figure 1:** Computational grid used in this work based on a fluid mesh.

**Figure 2:** Measurement points inserted into the radiation therapy ward configuration for the purpose of analyzing environmental parameters.

**Figure 3:** The number of measurement points that meet the suitable temperature and air flow speed range under eight conditions.

**Figure 4:** The average temperature of the four altitudes under eight conditions.

**Figure 5:** Average wind speed at four heights under eight conditions.

**Figure 6:** Airflow performance comparison.

**Figure 7:** Multidrug-resistant bacteria concentration distribution under different injection speeds based on (a) horizontal transmission line and (b) vertical transmission line.

**Figure 8:** Simulation of the spread of multidrug-resistant bacteria to different numbers of occupants based on variable ventilation speed in one directional air flow, where (a), (b), (c), and (d) describing the wind speed are equal to 5 m/s, 15 m/s, 25 m/s, and 35 m/s, respectively.

**Figure 9:** Simulation of the spread of multidrug-resistant bacteria in an occupated radiation therapy ward with nearly 200 people at every time step from *t* = 0 to *t* = 5.

**Table 1:** Specific characteristics of the eight situations.

Condition	Air volume (m^3^/h)	Air supply angle (°)
Situation 1	12,000	45
Situation 2	12,000	60
Situation 3	11,000	45
Situation 4	11,000	60
Situation 5	10,000	45
Situation 6	10,000	60
Situation 7	14,000	45
Situation 8	14,000	60

## Data Availability

Data is available on request from the authors due to privacy/ethical restrictions.
